This article has been retracted.

# Review of Brucellosis in Nepal

**DOI:** 10.4178/epih.e2016042

**Published:** 2016-10-01

**Authors:** Krishna Prasad Acharya, Nirajan Niroula, Krishna Kaphle

**Affiliations:** Institute of Agriculture and Animal Science, Tribhuwan University, Chitwan, Nepal

**Keywords:** Brucellosis, Zoonotic potential, Surveillance, Nepal

## Abstract

**OBJECTIVES:**

The aim of this paper is to evaluate the current status of the disease, the mechanism of infection, and pathogenesis, its zoonotic potential, diagnostic advances, treatment regimens, and the preventive measures that can be adopted in managing human brucellosis in under-developed countries such as Nepal.

**METHODS:**

We performed a systematic review of all the available literture through Google Scholar, PubMed, Gideon Informatics, World Health Organization and other legitimate sources. Other secondary informations were collected from the government agencies such as department of livestock services and Ministry of Health. The obtained information was then re-analysed and summarized.

**RESULTS:**

Few publications have addressed brucellosis in Nepal and most of those publications have focused on bovine brucellosis with sparse information available on brucellosis in humans and small ruminants. *Brucella abortus* is the most predominant causative agent followed by *B. suis. B. abortus* is predominant in cattle accounting for a substantial portion of bovine abortion in the country. Lack of awareness, unhealthy food habit, traditional husbandry practices, and a lack of surveillance and immunization have been the major factors in maintaining a vicious cycle of propagation of the disease in human and animals. Unfortunately, nothing has been done to identify the species of *Brucella* at the biovar level.

**CONCLUSIONS:**

Although brucellosis has been reported to be endemic in Nepal, neither the distribution nor the economic and public health impact of this disease is well characterized. Robust and well-designed nationwide survey is warranted to assess the prevalence and distribution of disease in livestock and humans. Such data would facilitate the design of appropriate control programmes.

## INTRODUCTION

Brucellosis is one of the important zoonotic diseases of livestock with worldwide distribution [1,2]. The most important brucellae of veterinary importance, and which cause abortion and infertility in female and male livestock are *Brucella abortus* (affecting bovines) *B. melitensis* (primarily affecting sheep and goats) and *B. suis* (primarily affecting pigs [2-4]. Establishment of the carrier state in animals can lead to a significant reduction in milk yield. This, together with losses through abortion or the early death of young offspring is a significant economic burden to farmers [5.6]. In regions where disease surveillance and control measures have not been implemented, long-term chronic infections are often associated with carpal hygromas and infertility [1,7].

The presentation of disease in male animals includes orchitis, epididymitis and seminal vesiculitis [4,6,8]. Brucellosis is a major public and animal health problem in areas with intensive, mixed types of farming, and where owners co-habit with their animals during the night [2,9,10]. In these systems, the mixed, migratory and free roaming nature of livestock herding makes it impractical to separate the diseased from healthy animals thus ensuring a favorable environment for *Brucella* transmission.

In Nepal, endemic bovine and caprine brucellosis pose a serious public health threat. Recent cases of human brucellosis in veterinary and para-veterinary students have been alarming serious. However, a systematic and large scale brucellosis control program targeting the eradication of the disease has not been adopted in Nepal. Financial constraints, inadequate laboratory facilities, lack of compliance by farmers, and religious taboos may impede the success of *Brucella* eradication in Nepal. Presently, the only control measures in place are those implemented voluntarily on a small number of commercial farms. Most livestock improvement approaches in Nepal are concentrated on the introduction of exotic animals, with a focus on up-grading and cross-breeding rather than on health. This disease has been given low priority by policy makers and hence limited resources have been allocated for the control of this disease. However, precise information on the distribution of brucellosis is absent and public health and economic impact of the disease have yet to be quantified. Objective data would allow rational decisions to be made regarding the best strategies and resource allocation for any control programs.

Although brucellosis has been widely reported in various species of animals and humans, only few studies have addressed this disease in the context of Nepal. Thus, the main purpose of this article is to thoroughly review the current literature and to propose guidelines suitable for Nepal.

## MAIN BODY

### Causative agent

Brucellosis is caused by infection with Gram-negative bacilli of the genus *Brucella*. The genus encompasses 10 recognized species including three species that are of major public health and economic importance [1]. These are *B. melitensis* which predominantly infects sheep and goats, *B. abortus* which affects cattle, and *B. suis,* which affects swine [1,9]. These species may also infect camelids, jacks and a variety of wildlife species. *B. melitensis,* *B. abortus*, and *B. suis* can be further sub-divided into biovars based on the unique phenotypic characteristics of different strains. Sub-species genotyping is also possible using molecular tools for analysis of genetic structure of the strains that have been isolated.

### Transmission

Chronically infected cattle may shed the organism via milk and reproductive tract discharges [11-13], and can also vertically transmit infection to their new born calves, thereby continuing the transmission of the disease [1,14,15]. Aborted fetuses from infected animals contain huge numbers of infectious organisms, and if not properly disposed of they form a major source of contamination [16,17]. The pathogen is highly contagious and is easily spread by licking the infected, aborted materials, discharges and waste of infected animals [16,18,19]. Direct contact with infected animals and consumption of contaminated dairy products may cause infection in human beings [20,21]. Human to human transmission is relatively uncommon [22]; however, it had been reported to occur after bone marrow transplantation [23,24], sexual intercourse [22], and blood transfusions [25]. Animals in Nepal are often housed in unhygienic sheds with poor management systems and also in close association with eachother (some sharing the same buildings). This presents a significant risk for the contraction of brucellosis in humans. Similarly, the consumption of raw milk, liver, spleen, udder, kidney, testis as well as handling of dung, which is widely prevalent in Nepal, may also be risk factors. Cultural practices such as consumption of raw yak blood during festivals may also pose a threat, but this has yet to be studied.

### Pathogenesis and immune response

The ability of the pathogen to survive and replicate within different host cells explains its pathogenicity [2,26,27]. Pathogenesis depends upon various factors such as the species, size of the inoculum, modes of transmission and the immune status of the host [28]. Extensive replication in placental trophoblasts is associated with abortion [1,28,29], and persistence in macrophages and other cell types leads to chronic infections [11,30, 31]. Protective immunity to the host is conferred by T-cell mediated macrophage activation by the antigenic protein of Brucella and the production of corresponding antibody along with other elements of immune response such as tumor necrosis factor (TNF), interferons and complement. Following infection, the immunoglobulin M (IgM) titer increases initially followed by the immunoglobulin G (IgG) titer. Thus, the apperance of IgM indicates an early immune response against brucellosis and IgG correspondingly indicates chronic infection or relapse [32,33].

### Global situation

Brucellosis is the second most important zoonotic disease in the world after rabies according to the World Organization for Animal Health. This disease is closely associated with the evolution of mankind as an agranian society and is linked to the practice of shepherding and popularization of animal husbandry. Brucellosis is widely prevalent throughout the world with the exception of northern, western and central parts of Europe, some Asian and American countries, Australia, and New Zealand [9,31,34]. At present, the global burden of brucellosis ranges from 1 to 200 new human cases per 10 millions individuals per year [34,35]. According to the available data, the incidence of human brucellosis is increasing in Eastern Mediterranean countries [36] and is endemic in some Asian countries including Sri Lanka [37], India [38], China [39], Pakistan [40], Mongolia [41], and Nepal [42-44]. Eradication of *Brucella* is feasible only if sufficient funds are available in the long term as well as well organized veterinary and public health services, coupled with a strong political will. However, most efforts have been abandoned due to lack of above mentioned conditions [2,45]. The prevalence of both animal and human brucellosis is significant in rural nomadic communities in many countries, including Nepal. *B. abortus* is the major species responsible for brucellosis in animals in some endemic countries, but due to the relatively low pathogenicity of *B. abortus* in humans, it is possible that many human cases go undetected. Thus, the low pathogenecity of *B. abortus* in humans and/or the low level of disease surveillance and monitoring could be possible causes of relatively low human incidence that has been reported in the endemic areas of the world.

### Current situation in Nepal

Few publications have addressed brucellosis in Nepal and most of those publications have focused on bovine brucellosis with sparse information available on brucellosis in humans and small ruminants. *B. abortus* is the most predominant causative agent followed by *B. suis*. *B. abortus* is predominant in cattle accounting for a substantial portion of bovine abortion in the country. Unfortunately, nothing has been done to identify the species of *Brucella* at the biovar level.

Although brucellosis has been reported to be endemic in Nepal, neither the distribution nor the economic and public health impact of this disease is well characterized [44,46]. Robust and well-designed nationwide survey is warranted to assess the prevalence and distribution of disease in livestock and humans. Such data would facilitate the design of appropriate control programmes.

### Brucellosis in animals

The presence of brucellosis in Nepal was first reported in 1977 by Pyakurel & Mishra [47]. Since then it has been reported in various parts of Nepal (Table 1) [48-53]. Pyakurel and Mishra [47] studied the sero-epidemiology of brucellosis in animals within Nepal and reported the highest prevalence (22.64%) in buffaloes from Pokhara. In another study carried out by Joshi reported a prevalence of 6.08% in humans, 8.70% in cattle, and 3.64% in sheep and goats [48]. The Department of Health Service reported that approximately 2% to 3% of cattle in Nepal are sero-positive for brucellosis based on nationwide surveys. The published reports, including the recent findings indicate that human and animal brucellosis is quite common in Nepal [44,47]. The seroprevalence of brucellosis has been found to vary across species of animals (17.60% in yak, nak and chauri, 10% in dogs, 8.70% in cattle and buffaloes, 3.64% in sheep and goats, and 7.18% in pigs) and also across regions (1.49% to 5.36%) with highest number of cases found in Solukhumbu (5.36%) and the lowest in Pokhara (1.49%). In cold places such as Solukhumbu, animals are housed in close space with high stocking density which could facilitate the transmission of infection.

From the period of 2003 to 2013, the Central Veterinary Laboratory [54] used the Rose Bengal Plate test (RBPT) to test 5,057 representative serum samples of cattle, buffalo, sheep and goat that were suspected to have brucellosis. The reported sero-positivity was 1.48%. Adhikari [55] reported 2% sero-positivity in goats from Dang, with females having a higher prevalence than males. The higher prevalence rate in females than their male counterparts could be attributed to the maternal behaviour to lick their infected newly born calves which can lead to re-infection. Similarly, the variation in prevalence between the sexes could have been due to the inherent variabilities, including physiological and behavioural factors. In a recent study by Pandey et al. [45], 32% of cattle, 13.40% of buffaloes, and 2.60% goats were found to be sero-positive when tested by plate agglutination test (PAT). Brucellosis is endemic and is increase in prevalence due to changes in the farming practices, increased movements and increased trade of animals [56]. It was suggested by Mantur & Amarnath [57] that widespread use of bulls for natural insemination might be a factor for contributing to widespread nature of brucellosis in cattle in Nepal. Unlike India and other countries of the world, a religious taboo on slaughtering of cattle may also have contributed to widespread distribution of bovine brucellosis in Nepal. Additionally, a free grazing system, sharing of breeding stock, and the frequent mixing of animals of different species may also have played a role in fostering a favorable environment for the spread of *Brucella* in Nepal.

### Brucellosis in humans

Brucellosis is a significant public health problem in Nepal. The first human case was reported in 1979 when the disease was diagnosed by the isolation of *B. melitensis* in a shepherd from Pokhara, who most likely acquired the disease from his sheep (Table 2). As recorded by various studies [59,61-64], have found prevelance of brucellosis in Nepalese males to be 5.60% to 9.42%, and 2.90% to 60% in females. Joshi et al. [58] conducted a repeated study on human brucellosis, and found its prevalence to be 4.48%. Joshi et al. [56] reported the occurrence to be 1.4% in human, which is lower than the finding of Singh [61], who reported a prevalence of 11.7% in workers of an abattoir in Kathmandu Valley (Table 2). This higher incidence of brucellosis among slaughterhouse workers may have been due to occupational exposure and poor hygiene in slaughterhouses. Aryal [64] reported the sero-prevalence of human brucellosis in Kathmandu to be 11.93%, and Jackson et al. [44] likewise reported widespread sero-positivity of *brucella* in both humans and Yak in Dolpa. In total, 84 cases of human brucellosis have been confirmed by serology with positive clinical signs from 1991 to 1997 [58] as well as 112 confirmed positive cases of human brucellosis between 1997 and 2002 [64]. Three major species of brucellosis (*B. abortus*, *B. melitensis*, and *B. suis*) have been reported to be present, although the precise distribution and prevalence of human brucellosis has yet to be determined [64]. In Nepal, approximately 90% of people live in villages and come into direct contact with domestic animals on a daily basis [47]. As a consequence, the local people of the villages are at a high risk of acquiring these types of zoonotic diseases [61,64]. Brucellosis has been found to vary by occupation (6.08% to 11.7%) and abattoir workers may be more at risk due to occupational exposure. The higher sero-positivity in males than in females might be due to male having closer contact with animals, and greater mobility [64]. The overall prevalence of brucellosis was 110 cases/10,000 inhabitants, which decreased to less than 20 cases/10,000 inhabitants from 2003 onwards [65]. This reduction in reported cases of brucellosis from 2003 onwards may have either been due to a lack of disease surveillance, resulting from the under-reporting of the disease in Nepal, or an increased awareness among veterinary practitioners and farmers. Moreover, the control of dairy products and changes in their production (such as compulsory pasteurization of products for public consumption) may be another possible reason for these observations.

### Clinical symptoms in humans

The clinical presentation of brucellosis is non-specific and requires laboratory testing for confirmation. Common presentations include fever, nausea, anorexia, headache, sweating, and prostration and these symptoms can be coupled with gastro-intestinal, musculoskeletal, hepato-biliary and meningeo-vascular complications [31]. Fever is the most common manifestation followed by arthritis, sweating and constitutional symptoms [34,67-69]. It may appear as acute, with an incubation period of two to three weeks or in a sub-acute or chronic form with an incubation period of weeks to months.

### Diagnosis

Brucellae are intra-cellular pathogens in cells of the immune system and therefore difficult to diagnose and treat. The definitive diagnosis requires the isolation of the organism from the patient, but is restricted by the fact that *Brucella* spp. are slow-growing intracellular pathogens, the successful culture of which from blood decreases as the disease progresses [70,71]. The previous use of antibiotics also adds to the difficulty of culturing the bacillus [72]. As such, successful diagnosis necessitates a careful selection of the best suitable culture method and validation of its performance. The sensitivity of culturing *Brucella* spp. from blood varies from 15% to 70% as assessed in reference to clinical evidence of infection and positive serological results depending on the study and culture method used [71].

Culture provides direct evidence of the presence of the pathogen and is the gold standard, but in the absence of adequate culture facilities, brucellosis can be diagnosed by serological testing. A variety of serological tests are available for the serodiagnosis of human brucellosis including the RBPT, the PAT, Serum agglutination test (SAT), 2-mercaptoethanol (2-ME), Coombs and enzyme linked immunosorbent assay (ELISA) tests. Most of the serological tests are highly sensitive, but are not quite specific. Different types of Gram-negative bacteria such as *Escherichia coli, Vibrio cholerae, Escherichia hermanni, Salmonella*, and *Francisella tularensis* elicit antibody responses that crossreact with Brucella antigen thus yielding low specificity. Although modern diagnostic techniques with high sensitivity and specificity, such as polymerase chain reaction (PCR) have been introduced, they are currently not widely used in field conditions.

The diagnosis of brucellosis in field conditions relies heavily on serological tests. However, specificity of such tests has been a major concern. As the specificity of these tests is less than 100% the interpretation of test results should be supplemented with the case history, clinical manifestation and other laboratory findings [73-75]. It is recommended to use at least two serological tests to confirm active infection in animals and humans.

The RBPT is the most commonly used agglutination test in diagnosis of brucellosis in field condition in which it is not possible to perform the SAT. The results of RBPT should always be confirmed by other tests due to its low sensitivity in chronic cases and low specificity in endemic areas [76].

In areas where the SAT can be used, it is usually used first followed by the 2-ME test to confirm the result of the SAT by excluding the possibility of cross reacting IgM antibodies. The result of 2-ME can sometimes be mis-interpreted in patients with low levels of IgG [77-81].

Specific IgM antibodies detected by ELISA are useful in diagnosis of acute brucellosis [73,82], whereas the Coombs test and IgG ELISA are useful for detecting of chronic infection and monitoring relapsing strains due to their ability to detect incomplete antibodies [82]. However, the dipstick test can be used in patients as a rapid and simple alternative to ELISA IgM test for the serodiagnosis of patients with acute brucellosis [83,84]. For the accurate diagnosis of a suspected case, a combination of ELISA IgM and IgG tests with follow-up and monitoring by ELISA IgM and 2-MET may be helpful due to promising efficiency of these tests [85]. In addition, fluorescence polarization assay (FPA) and immunocapture agglutination for anti-*Brucella* might be alternative choices due to their ability to detect the disease in patients with a longstanding evolution of brucellosis. *Brucella* IgM and IgG lateral flow [73] and latex agglutination [86,87] assays have also been found to be rapid and simple. Such techniques along with culturing suspected cases may prove useful for the field condition in remote areas where other methods may not be feasible.

Although the gold standard is the isolation of *Brucella* organism from blood and bone marrow, PCR based testing method is a more accurate one for testing the presence of *Brucella*, and promises to be a more useful and practical approach than culture [88]. PCR is particularly useful in patients with specific complications, such as neurobacillosis or other localized conditions not detectable using serological tests [89,90]. However, the quality control remains a matter of concern [3,91,92]. Overcoming drawbacks of conventional PCR, real time PCR has emerged as technique that is less prone to contamination, faster and clinically more useful [93,94]. However, the expensive nature of real time PCR has restricted its use in field conditions and in some developing countries

In summary, the presumptive diagnosis of brucellosis should be based on the patients’ history and clinical findings. These clinical findings should be combined with the RBPT or SAT, and positive reactions should be confirmed by additional confirmatory tests. In particular, positive results from a test involving detection of agglutinating antibodies (RBPT; SAT) should be combined with the test involving detection of non-agglutinating antibodies, such as ELISA or the Coomb’s test.

### Treatment of brucellosis

The treatment of brucellosis in animals is not effective, and infected animals should be isolated to prevent further transmission. If feasible, infected animals should be destroyed and properly disposed of. However, multi-drug regimens could be tried [69,95,96]. Treatment failure and relapse rates can be high and depend on the drug combination and compliance [69]. Despite several studies on the use of antibiotics for the management of brucellosis, no conclusive evidence supporting an optimal strategy for antimicrobial therapy has been reported [69,96]. The treatment for acute brucellosis recommended by the world health organization is oral doxycycline (100 mg twice a day) and oral rifampin (600 to 900 mg/d) for 6 weeks [97], but this regimen is not to be followed in cases complicated by spondylitis and tuberculosis due to the possibility of resistant *Mycobacterium tuberculosis* [98,99]. Rifampin mono-therapy is the primary choice for treating brucellosis during pregnancy and a combination of sulphamethoxazole and trimethoprim is used to treat brucellosis in children [100]. Clinical trials with other antibiotics such as quinolones, macrolides, sulpha-trimethoprim, cotrimoxazole and rifampin have resulted in poor results. Some localized forms of brucellosis such as endocarditis, meningitis and spondylitis should be treated through surgery supplemented by triple antibiotic therapy (doxycycline, rifampicin, and trimethoprim-sulfamethoxazole) [101]. The antibiotic regimen must be selected based on patients’ underlying conditions and the location of the disease [102-105]. In Nepal, although it has been reported to be endemic, animals are abandoned rather than treated.

### Measures for controlling brucellosis in animals and humans

In absence of human vaccines, the control of human brucellosis is achievable through control of the disease in animals. Brucellosis in animals may be controlled by the strict enforcement of a set of measures including testing and slaughtering, vaccination, sanitation, and movement control [31]. However, the control of brucellosis has proven to be cumbersome in Hindu-dominated countries such as Nepal, as the slaughtering of cattle is prohibited. Knowledge of the distribution and spread of brucellosis and its presence in the different livestock and wildlife species is essential for the effective implementation of control measures. A few serological studies have investigated the presence and distribution of brucellosis in livestock and humans in Nepal and the risk of transmission to the human population.

The lack of awareness among farmers, and the absence of an effective control strategy have made the situation favorable for the endemicity of brucellosis in Nepal. Thus, animal owners should be made aware of the economic, and health impact of brucellosis and the importance of vaccinating their livestock. Public health education should emphasize food and occupational hygiene. Avoiding or discouraging the consumption of raw milk and dairy products as well as a strict procedure involving protective and safety measures among health workers will help prevent brucellosis in the human population. Rev1, a modified live bacterial vaccine can be used in small ruminants at three to four months of age providing immunity for three to five years. Strain 19 and RB51 are commonly used for the prevention of brucellosis in cattle. These vaccines are used to vaccinate calves between four to twelve months of age. The latter is more advantageous because the immunity induced by RB51 is less abortogenic and is non-complex, meaning that serological findings in infected animals can be easily differentiated from those of vaccinated animals.

## RECOMMENDATIONS

### Increase public awareness

Efforts should be made by the government and the other concerned parties to raise awareness of the disease and its impact on public health. The first weapon of disease prevention is the minimization of exposure, which can be achieved by educating the high risk groups including farmers, and members of similar occupational categories. Protective clothing and other protective measures should be used during handling of animals. Training should be provided for farmers and livestock attendants regarding effective sanitary and hygienic management practices during handling of animals and animal products such as aborted fetal materials and other body secretions. Thus, in under-developed countries like Nepal, where the elimination of infected animals is not feasible, prevention of human infection should be grounded in principles of public awareness, food safety measures, and occupational hygiene.

### Food hygiene

Since *Brucella* is readily killed by heat treatment, boiling milk and heating milk products to 80-85 degrees centigrade make them safe for human consumption. Cultural practices like drinking milk directly from the udder, as well as using uncooked cow milk and urine to make elixirs should be carefully studied to assess their likelihood of resulting in an infection. Research is also required to determine whether cultural practices such as drinking raw yak blood pose a risk for transmission of brucellosis.

### Control of brucellosis in animals by regular surveillance, screening and immunization

Regular surveillance is necessary as it is one of the important steps in preventive and control measures. Cost-effective surveillance method includes regular testing of bulk quantities of milk [1], and using the RBPT, and PAT test to screen for positive animals. Although the milk ring test is not effective test for testing the milk of sheep and goats due to its fatty nature, other alternatives such as the RBPT and PAT can be used effectively [1]. The strict implementation of quarantine and sero-surveillance is an utmost necessity [1]. Detailed epidemiological investigation of the three pillars of the disease should be conducted across the country to identify the risk factors with the occurrence and endemicity of disease. The immunization of animals with vaccines is of utmost importance for prevention and control efforts [11,106-111].

### Maintaining healthy contact with animals

Since the sharing of water points for drinking and grazing lands are important risk factors for transmission of brucellosis, avoiding the mixing of cattle and other animals as well as raising replacement heifers within a herd might be important steps in the control and prevention of brucellosis in humans and animals. Screening animals before purchasing and incorporating them into a herd, the proper disposal of aborted materials and the isolation of animals during parturition would help to reduce the transmission of brucellosis across the herd [108].

### Testing and slaughtering of infected animals

Testing and slaughtering can be a cost effective method of control [7,106]. In Nepal, the test and slaughter method is difficult due to the high cost involved in the slaughter of animals [109,112,113] and the religious taboo against slaughtering cattle. The control of disease in animals in Nepal should depend on the mass vaccination of all animals for the first few years until the incidence of infection declines up to 1% or even lower. The test and slaughter method can then be used, because it will be non-expensive. Moreover, full cooperation of the government and other stakeholders will be necessary for this method to be successful.

## CONCLUSION

As in other under-developed and developing countries of world, the situation involving brucellosis is alarmingly serious in Nepal. Extensive research on the epidemiology and public health impacts of brucellosis is urgently necessary. Efforts should be made to control brucellosis in animals and to reduce its transmission to human. Vaccination and awareness program should be strengthened by veterinary and para-veterinary services. In rural Nepal, knowledge about basic food safety and disease transmission is lacking. Small, simple changes based on the identification of risk are likely to make a large impact.

## Figures and Tables

**Table 1.** Seroprevalence of brucellosis in animals in Nepal

District	Species	No. of tested animals	No. of positive animals (%)	Reference	
Solukhumbu	Yak and Nak	31			
Jumla	Yak, Nak, Chauri, Cattle	95	16 (16.84)	Pyakurel & Mishra [47]	
Kathmandu	Cattle, Pigs, Goats	146	26 (17.47)		
Kaski	Buffaloes	53	12 (22.64)		
Chitwan	Sheep and Goats	24	4 (16.67)		
Biratnagar	Cattle	72	1 (1.38)		
	Cattle				
Chitwan	Cattle and Buffaloes	1,069	93 (8.7)	Joshi [48]	
	Sheep and Goats	247	9 (3.6)		
Kathmandu	Cattle	120	15 (12.5)	Joshi [58]	
Chitwan	Sheep	14	2 (14.3)	Joshi et al. [59]	
Chitwan	Dairy cows	91	3 (3.4)	Pradhan [50]	
Langtang valley	Yak, Chauri and hilly cattle	74	13 (17.6)	Lefkowitz et al. [53]	
Chitwan	Goats	56	3 (5.4)	Dhakal et al. [60]	
	Buffaloes	35	1 (2.9)		
Kathmandu	Buffaloes	153	0 (0.0)	Shrestha [62]	
	Pigs	153	11 (17.1)		
	Goat	70	12 (7.2)		
Kathmandu	Pigs	190	41 p1.6)	Rana [51]	
Makawanpur	Goats	41	12 (29.3)		
Chitwan	Goats	39	2 (5.1)		
	Sheep	12	2 (14.3)	Poudel [55]	
Kathmandu	Goats	37	2 (5.4)		
Kailali	Cattle	50	16 (32.0)	Pandey et al. [45]	
	Buffaloes	67	9 (13.4)		
	Goats	116	3 (2.6)		
Taplejung & Lumjung	Goats	139	24 (17.3)	Das et al. [49]	
	Sheep	246	55 (22.3)		

**Table 2.** Seroprevalence of brucellosis in humans in Nepal

Location	Patient types	Test employed	Prevalence (%)	References	
Kathmandu	Indoor and outdoor patients	PAT, SAT, 2-ME	57/2,117 (2.7)	Joshi et al. [63]	
	Patients admitted to Bir Hospital	SAT	28/200 (14.0)	Rana [43]	
Kathmandu		SAT	87/1,430 (6.1)	Joshi [48]	
Kathmandu	Humans of Kathmandu valley	PAT	3/121 (2.5) 3/5,000 (0.1)	Pyakurel & Mishra [47]	
		PAT	120/1,006 (11.9)	Singh [61]	
	General population	PAT	25/558 (4.5)	Aryal [64]	
		PAT	123/1,506 (8.2)	Joshi [56]	
	Patients showing the one or more symptoms of brucellosis	PAT	1 case	Joshi et al. [64]	
Pokhara	Sheep herders	PAT, ELISA		Dickenson & Thaller [66]	

PAT, plate agglutination test; SAT, serum agglutination test; 2-ME, 2-mercaptoethanol test; ELISA, enzyme linked immuno-sorbent assay.

## References

[1] World Health Organization (2006). Brucellosis in humans and animals.

[2] Muflihanah H, Hatta M, Rood E, Scheelbeek P, Abdoel TH, Smits HL (2013). Brucellosis seroprevalence in Bali cattle with reproductive failure in South Sulawesi and Brucella abortus biovar 1 genotypes in the Eastern Indonesian archipelago. BMC Vet Res.

[3] Nimri LF (2003). Diagnosis of recent and relapsed cases of human brucellosis by PCR assay. BMC Infect Dis.

[4] Cutler SJ, Whatmore AM, Commander NJ (2005). Brucellosis--new aspects of an old disease. J Appl Microbiol.

[5] Smits HL, Kadri SM (2005). Brucellosis in India: a deceptive infectious disease. Indian J Med Res.

[6] Schelling E, Diguimbaye C, Daoud S, Nicolet J, Boerlin P, Tanner M (2003). Brucellosis and Q-fever seroprevalences of nomadic pastoralists and their livestock in Chad. Prev Vet Med.

[7] Refai M (2002). Incidence and control of brucellosis in the Near East region. Vet Microbiol.

[8] Agasthya AS, Isloor S, Prabhudas K (2007). Brucellosis in high risk group individuals. Indian J Med Microbiol.

[9] Armon L, Hadani Y, Chechik C, Bardenstein S (2015). Large human Brucella melitensis outbreak in Israel, 2014. Isr J Vet Med.

[10] Jones BA, Grace D, Kock R, Alonso S, Rushton J, Said MY (2013). Zoonosis emergence linked to agricultural intensification and environmental change. Proc Natl Acad Sci U S A.

[11] Nielsen K, Duncan JR (1990). Animal brucellosis.

[12] Abubakar M, Javed Arshed M, Hussain M, Ehtisham-ul- Haq, Ali Q (2010). Serological evidence of Brucella abortus prevalence in Punjab province, Pakistan--a cross-sectional study. Transbound Emerg Dis.

[13] Nikokar I, Hosseinpour M, Asmar M, Pirmohbatei S, Hakeimei F, Razavei MT (2011). Seroprevalence of Brucellosis among high risk individuals in Guilan, Iran. J Res Med Sci.

[14] Magableh SM, Bataineh HA (2007). Clinical study of childhood brucellosis in Jordan. Middle East J Fam Med.

[15] Kato Y, Masuda G, Itoda I, Imamura A, Ajisawa A, Negishi M (2007). Brucellosis in a returned traveler and his wife: probable person-to-person transmission of Brucella melitensis. J Travel Med.

[16] Deqiu S, Donglou X, Jiming Y (2002). Epidemiology and control of brucellosis in China. Vet Microbiol.

[17] Pappas G, Bosilkovski M, Akritidis N, Mastora M, Krteva L, Tsianos E (2003). Brucellosis and the respiratory system. Clin Infect Dis.

[18] Muma JB, Samui KL, Siamudaala VM, Oloya J, Matop G, Omer MK (2006). Prevalence of antibodies to Brucella spp. and individual risk factors of infection in traditional cattle, goats and sheep reared in livestock-wildlife interface areas of Zambia. Trop Anim Health Prod.

[19] Matope G, Bhebhe E, Muma JB, Lund A, Skjerve E (2010). Herd-level factors for Brucella seropositivity in cattle reared in smallholder dairy farms of Zimbabwe. Prev Vet Med.

[20] Olsen S, Tatum F (2010). Bovine brucellosis. Vet Clin North Am Food Anim Pract.

[21] Ducrotoy MJ, Bertu WJ, Ocholi RA, Gusi AM, Bryssinckx W, Welburn S (2014). Brucellosis as an emerging threat in developing economies: lessons from Nigeria. PLoS Negl Trop Dis.

[22] Mantur BG, Mangalgi SS, Mulimani M (1996). Brucella melitensis--a sexually transmissible agent?. Lancet.

[23] Ertem M, Kürekçi AE, Aysev D, Unal E, Ikincioğullari A (2000). Brucellosis transmitted by bone marrow transplantation. Bone Marrow Transplant.

[24] Arenas GN, Staskevich AS, Aballay A, Mayorga LS (2000). Intracellular trafficking of Brucella abortus in J774 macrophages. Infect Immun.

[25] Economidou J, Kalafatas P, Vatopoulou T, Petropoulou D, Kattamis C (1976). Brucellosis in two thalassaemic patients infected by blood transfusions from the same donor. Acta Haematol.

[26] Ray K, Marteyn B, Sansonetti PJ, Tang CM (2009). Life on the inside: the intracellular lifestyle of cytosolic bacteria. Nat Rev Microbiol.

[27] Alavi SM, Motlagh ME (2012). A review of epidemiology, diagnosis and management of brucellosis for general physicians working in the Iranian health network. Jundishapur J Microbiol.

[28] Djønne B (2007). Infections and perinatal diseases: a comparative overview. Acta Vet Scand.

[29] Rodríguez MC, Viadas C, Seoane A, Sangari FJ, López-Goñi I, García-Lobo JM (2012). Evaluation of the effects of erythritol on gene expression in Brucella abortus. PLoS One.

[30] Gilbert P, Holst F, Rossbach J, Pauli HK (1991). Brucellosis-induced granulomatous non-puerperal mastitis--a case report. Geburtshilfe Frauenheilkd.

[31] Pappas G, Papadimitriou P, Akritidis N, Christou L, Tsianos EV (2006). The new global map of human brucellosis. Lancet Infect Dis.

[32] Young EJ, Mandell GL, Douglas RG, Bennett JE, Dolin R (2005). Brucella species. Mandell, Douglas, and Bennett’s principles and practice of infectious diseases.

[33] McDonald WL, Jamaludin R, Mackereth G, Hansen M, Humphrey S, Short P (2006). Characterization of a Brucella sp. strain as a marine-mammal type despite isolation from a patient with spinal osteomyelitis in New Zealand. J Clin Microbiol.

[34] Dean AS, Crump L, Greter H, Hattendorf J, Schelling E, Zinsstag J (2012). Clinical manifestations of human brucellosis: a systematic review and meta-analysis. PLoS Negl Trop Dis.

[35] Minas M, Minas A, Gourgulianis K, Stournara A (2007). Epidemiological and clinical aspects of human brucellosis in Central Greece. Jpn J Infect Dis.

[36] Hegazy YM, Ridler AL, Guitian FJ (2009). Assessment and simulation of the implementation of brucellosis control programme in an endemic area of the Middle East. Epidemiol Infect.

[37] Priyantha MA (2011). Identification of biovars of Brucella abortus in aborted cattle and buffaloes herd in Sri Lanka. Vet World.

[38] Ghodasara SN, Roy A, Bhanderi BB (2010). Comparison of Rose Bengal plate agglutination, standard tube agglutination and indirect ELISA tests for detection of Brucella antibodies in cows and buffaloes. Vet World.

[39] Deqiu S, Donglou X, Jiming Y (2002). Epidemiology and control of brucellosis in China. Vet Microbiol.

[40] Akhtar R, Chaudhry ZI, Shakoori AR, Ahmad MU, Aslam A (2010). Comparative efficacy of conventional diagnostic methods and evaluation of polymerase chain reaction for the diagnosis of bovine brucellosis. Vet World.

[41] Zinsstag J, Roth F, Orkhon D, Chimed-Ochir G, Nansalmaa M, Kolar J (2005). A model of animal-human brucellosis transmission in Mongolia. Prev Vet Med.

[42] Knox C, Gillies L, Joshi DD (2000). Veterinary public health in the Nepal Himalaya. Can Vet J.

[43] Rana HB (2002). Sero-epidemiological surveillance of Human and Animal Brucellosis in Surkhet District, Mid-western Region of Nepal. M. Sc. Zoology Thesis.

[44] Jackson DS, Nydam DV, Altier C (2014). Prevalence and risk factors for brucellosis in domestic yak Bos grunniens and their herders in a transhumant pastoralist system of Dolpo, Nepal. Prev Vet Med.

[45] Pandeya YR, Joshi DD, Dhakal S, Ghimire L, Mahato BR, Chaulagain S (2013). Seroprevalence of brucellosis in different animal species of Kailali district, Nepal. Int J Infect Microbiol.

[46] Aryal S, Paudel KP (2007). Reproductive disorders and seroprevalence of brucellosis in Yak. Nepal Agric Res J.

[47] Pyakural S, Mishra U (1977). Sero-epidemiological evidence of animal brucellosis in Nepal. Bull Vet Sci Anim Husb Nepal.

[48] Joshi DD (1983). A Public Health problem in Nepal. Bulletin of Veterinary Science and Animal Husbandry Nepal.

[49] Das LN, Singh S, Singh UM, Singh DK (2016). Prevalence of brucellosis in migratory sheep and goat of Taplejung and Lamjung District, Nepal. Nepalese Vet J.

[50] Pradhan A (1996). Sero surveillance of brucellosis in cattle and buffaloes in Chitwan.

[51] Rana S (2005). Seroprevalence of Brucellosis in Slaughter Swine in the Kathmandu valley. B.V.Sc & AH internship report IAAS.

[52] Paudel A (2006). Seroprevalence of Brucellosis in Small ruminants in Nepal. B.V.Sc & AH internship report IAAS.

[53] Lefkowitz NA, Joshi DD, Chhetri DB, Sharma M (2003). Prevalence of Brucellosis in Yak and Other Cattle of Langtang Valley. Nepalese Vet.J.

[54] CVL (VEC) (2012). Annual Epidemiological Bulletin-2005, (Jan.–Dec.). Veterinary Epidemiology Center, Directorate of Animal Health, Tripureswor.

[55] Adhikari S (2012). Prevalence of brucellosis in goats of Dang districts, Nepal Souenir 2012.

[56] Joshi DD (2000). Epidemiological Surveillance of Human and Animal Brucellosis in Milk collection area of DDC, Nepal.

[57] Mantur BG, Amarnath SK (2008). Brucellosis in India - a review. J Biosci.

[58] Joshi DD (1992). Status of brucellosis in man and animals in Nepal, WHO/SEARO.

[59] Joshi DD, Upadhya M, Mishra PN (2005). Brucellosis in animal and human of Chitwan NZFHRC Tahachal.

[60] Jost CC, Dhakal LP, Regmi TR, Joshi DD (2005). Training communities in livestock-derived food safety and hygiene in Chitwan district, Nepal.

[61] Singh HL (1985). Principal records of Nepal: a collection of important facts and events of Nepal in the chronological order.

[62] Shrestha B (2008). Sero-prevalence of Brucellosis in different species of meat animals of Nepal. B.V.Sc & AH internship report. IAAS.

[63] Joshi DD (1984). Incidence of human brucellosis in Kathmandu. JNMA J Nepal Med Assoc.

[64] Joshi DD, Shrestha IL, Aryal A (2007). Veterinary and human public health importance of brucellosis in Nepal. Nepal Vet J.

[65] Berger SA (2014). Infectious diseases of Nepal.

[66] Dickenson JG, Thaller VT (1979). Brucellosis in shepherds in Nepal. JNMA J Nepal Med Assoc.

[67] Bukharie HA (2009). Clinical features, complications and treatment outcome of Brucella infection: ten years’ experience in an endemic area. Trop J Pharm Res.

[68] Mantur BG, Akki AS, Mangalgi SS, Patil SV, Gobbur RH, Peerapur BV (2004). Childhood brucellosis--a microbiological, epidemiological and clinical study. J Trop Pediatr.

[69] Falagas ME, Bliziotis IA (2006). Quinolones for treatment of human brucellosis: critical review of the evidence from microbiological and clinical studies. Antimicrob Agents Chemother.

[70] Işeri S, Bulut C, Yetkin MA, Kinikli S, Demiröz AP, Tülek N (2006). Comparison of the diagnostic value of blood and bone marrow cultures in brucellosis. Mikrobiyol Bul.

[71] Alişkan H (2008). The value of culture and serological methods in the diagnosis of human brucellosis. Mikrobiyol Bul.

[72] Al-Tawfiq JA, Abukhamsin A (2009). A 24-year study of the epidemiology of human brucellosis in a health-care system in Eastern Saudi Arabia. J Infect Public Health.

[73] Smits HL, Abdoel TH, Solera J, Clavijo E, Diaz R (2003). Immunochromatographic Brucella-specific immunoglobulin M and G lateral flow assays for rapid serodiagnosis of human brucellosis. Clin Diagn Lab Immunol.

[74] Özdemir M, Feyzioğlu B, Kurtoğlu MG, Doğan M, Dağı HT, Yüksekkaya Ş (2011). A comparison of immuncapture agglutination and ELISA methods in serological diagnosis of brucellosis. Int J Med Sci.

[75] Fadeel MA, Hoffmaster AR, Shi J, Pimentel G, Stoddard RA (2011). Comparison of four commercial IgM and IgG ELISA kits for diagnosing brucellosis. J Med Microbiol.

[76] Mantur BG, Biradar MS, Bidri RC, Mulimani MS, Kariholu P (2006). Protean clinical manifestations and diagnostic challenges of human brucellosis in adults: 16 years’ experience in an endemic area. J Med Microbiol.

[77] El Sherbini A, Kabbash I, Schelling E, El Shennawy S, Shalapy N, Elnaby GH (2007). Seroprevalences and local variation of human and livestock brucellosis in two villages in Gharbia Governorate, Egypt. Trans R Soc Trop Med Hyg.

[78] Doyle TJ, Bryan RT (2000). Infectious disease morbidity in the US region bordering Mexico, 1990-1998. J Infect Dis.

[79] Christopher S, Umapathy BL, Ravikumar KL (2010). Brucellosis: review on the recent trends in pathogenicity and laboratory diagnosis. J Lab Physicians.

[80] Araj GF (2010). Update on laboratory diagnosis of human brucellosis. Int J Antimicrob Agents.

[81] Mantur B, Parande A, Amarnath S, Patil G, Walvekar R, Desai A (2010). ELISA versus conventional methods of diagnosing endemic brucellosis. Am J Trop Med Hyg.

[82] Pabuccuoglu O, Ecemis T, El S, Coskun A, Akcali S, Sanlidag T (2011). Evaluation of serological tests for diagnosis of brucellosis. Jpn J Infect Dis.

[83] Lim ML, Richman LS (2004). Brucellosis. Infect Dis Clin Pract (Baltim Md).

[84] Taleski V (2010). An overview of introducing various laboratory tests for diagnosis of human brucellosis in the Republic of Macedonia. Maced J Med Sci.

[85] Asaad AM, Alqahtani JM (2012). Serological and molecular diagnosis of human brucellosis in Najran, Southwestern Saudi Arabia. J Infect Public Health.

[86] Nielsen K Gall D (2001). Fluorescence polarization assay for the diagnosis of brucellosis: a review. J Immunoassay Immunochem.

[87] Abdoel TH, Smits HL (2007). Rapid latex agglutination test for the serodiagnosis of human brucellosis. Diagn Microbiol Infect Dis.

[88] Yu WL, Nielsen K (2010). Review of detection of Brucella spp. by polymerase chain reaction. Croat Med J.

[89] Colmenero JD, Queipo-Ortuño MI, Reguera JM, Baeza G, Salazar JA, Morata P (2005). Real time polymerase chain reaction: a new powerful tool for the diagnosis of neurobrucellosis. J Neurol Neurosurg Psychiatry.

[90] Newby DT, Hadfield TL, Roberto FF (2003). Real-time PCR detection of Brucella abortus: a comparative study of SYBR green I, 5’-exonuclease, and hybridization probe assays. Appl Environ Microbiol.

[91] Khosravi AD, Abassi E, Alavi SM (2006). Isolation of Brucella melitensis and Brucella abortus from brucellosis patients by conventional culture method and polymerase chain reaction technique. Pak J Med Sci.

[92] Gemechu MY, Gill JP, Arora AK, Ghatak S, Singh DK (2011). Polymerase chain reaction (PCR) assay for rapid diagnosis and its role in prevention of human brucellosis in Punjab, India. Int J Prev Med.

[93] Probert WS, Schrader KN, Khuong NY, Bystrom SL, Graves MH (2004). Real-time multiplex PCR assay for detection of Brucella spp., B. abortus, and B. melitensis. J Clin Microbiol.

[94] Debeaumont C, Falconnet PA, Maurin M (2005). Real-time PCR for detection of Brucella spp. DNA in human serum samples. Eur J Clin Microbiol Infect Dis.

[95] Roushan MR, Gangi SM, Ahmadi SA (2004). Comparison of the efficacy of two months of treatment with co-trimoxazole plus doxycycline vs. co-trimoxazole plus rifampin in brucellosis. Swiss Med Wkly.

[96] Al-Anazi KA, Al-Jasser AM (2014). Brucellosis: a global re-emerging zoonosis; diagnosis, treatment and prevention.

[97] Alp E, Koc RK, Durak AC, Yildiz O, Aygen B, Sumerkan B (2006). Doxycycline plus streptomycin versus ciprofloxacin plus rifampicin in spinal brucellosis [ISRCTN31053647]. BMC Infect Dis.

[98] Ariza J, Bosilkovski M, Cascio A, Colmenero JD, Corbel MJ, Falagas ME (2007). Perspectives for the treatment of brucellosis in the 21st century: the Ioannina recommendations. PLoS Med.

[99] Skalsky K, Yahav D, Bishara J, Pitlik S, Leibovici L, Paul M (2008). Treatment of human brucellosis: systematic review and meta-analysis of randomised controlled trials. BMJ.

[100] Khuri-Bulos NA, Daoud AH, Azab SM (1993). Treatment of childhood brucellosis: results of a prospective trial on 113 children. Pediatr Infect Dis J.

[101] Yilmaz E, Parlak M, Akalin H, Heper Y, Ozakin C, Mistik R (2004). Brucellar spondylitis: review of 25 cases. J Clin Rheumatol.

[102] McLean DR, Russell N, Khan MY (1992). Neurobrucellosis: clinical and therapeutic features. Clin Infect Dis.

[103] Alavi SM, Rajabzadeh AR (2007). Comparison of two chemotherapy regimen: doxycycline-rifampicin and doxycycline cotrimoxazol in the brucellosis patients Ahvaz, Iran, 2004-2006. Pak J Med Sci.

[104] Ersoy Y, Sonmez E, Tevfik MR, But AD (2005). Comparison of three different combination therapies in the treatment of human brucellosis. Trop Doct.

[105] Karabay O, Sencan I, Kayas D, Sahin I (2004). Ofloxacin plus rifampicin versus doxycycline plus rifampicin in the treatment of brucellosis: a randomized clinical trial [ISRCTN11871179]. BMC Infect Dis.

[106] Ragan VE, Animal and Plant Health Inspection (2002). The Animal and Plant Health Inspection Service (APHIS) brucellosis eradication program in the United States. Vet Microbiol.

[107] Russo G, Pasquali P, Nenova R, Alexandrov T, Ralchev S, Vullo V (2009). Reemergence of human and animal brucellosis, bulgaria. Emerg Infect Dis.

[108] Hotez PJ, Savioli L, Fenwick A (2012). Neglected tropical diseases of the Middle East and North Africa: review of their prevalence, distribution, and opportunities for control. PLoS Negl Trop Dis.

[109] Blasco JM, Molina-Flores B (2011). Control and eradication of Brucella melitensis infection in sheep and goats. Vet Clin North Am Food Anim Pract.

[110] Olsen SC, Stoffregen WS (2005). Essential role of vaccines in brucellosis control and eradication programs for livestock. Expert Rev Vaccines.

[111] Vemulapalli R, He Y, Sriranganathan N, Boyle SM, Schurig GG (2002). Brucella abortus RB51: enhancing vaccine efficacy and developing multivalent vaccines. Vet Microbiol.

[112] Rivera SA, Ramírez MC, Lopetegui IP (2002). Eradication of bovine brucellosis in the 10th Region de Los Lagos, Chile. Vet Microbiol.

[113] Havas KA (2012). A systemic review of brucellosis in the Kakheti region of the country of Georgia: An evaluation of the disease ecology, risk factors and suggestions for disease control [dissertation].

